# The Impact of Hearing Aids on Speech Perception in Mandarin-Speaking Children

**DOI:** 10.1155/2022/8692865

**Published:** 2022-08-12

**Authors:** Yuan Zhang, Yun Zheng, Gang Li

**Affiliations:** Department of Otolaryngology & Head and Neck Surgery, West China Hospital of Sichuan University, No. 37 Guo Xue Xiang, Chengdu, Sichuan 610041, China

## Abstract

**Background:**

Severe hearing loss can affect speech perception in children, and hearing aids as a medical device may help improve speech perception in children.

**Objective:**

To explore the effects of fitting hearing aids (HAs) on speech perception in children with severe hearing loss (60–70 dB HL).

**Methods:**

Ninety-five children with bilateral severe hearing loss who were fitted bilaterally with HAs before the age of 3 years were followed up. The subjects were grouped according to their age at the time of fitting, i.e., <1, 1–2 , and 2–3 years groups. The Mandarin Early Speech Perception test was used to evaluate speech perception of Mandarin monosyllabic words at 12, 24, and 36 months after fitting.

**Results:**

There were significant improvements in vowel, consonant, and tone perception scores from 12 to 36 months after fitting HAs in the three age groups, and the mean score at 36 months after fitting was significantly improved at >85%. The mean speech pattern and spondee perception scores averaged at >90% at 12 months after fitting and were comparable to the scores of 2-year-old children with normal hearing.

**Conclusions:**

HA helps with speech perception in children with severe hearing loss.

## 1. Introduction

Learning to speak strongly depends on speech perception, which is accurately perceiving and decoding speech signals [1]. The improvement of speech recognition indicates whether children with hearing loss (HL) have received effective intervention. The materials of speech perception are presented in open and closed sets. Closed-set speech perception tests require the children to choose from limited options, whereas there are unlimited choices in open-set tests. As open-set speech perception tests are closer to the real-world listening conditions to some extent, they are preferred over closed-set tests for assessing speech perception in children with HL.

In previous studies, for children with the same degree of HL, the difference in speech perception test results between children with hearing aids (HAs) and children with cochlear implants (CIs) formed the basis for determining the target population for CIs [2, 3]. Indications for CIs have expanded from profound to severe HL. Unlike children with profound bilateral HL for whom CIs can be confidently recommended based on an unaided audiogram, children with severe HL need a comprehensive evaluation of their speech and language development to make such a recommendation. Therefore, dynamic monitoring of the auditory and speech development of children with severe HL who have been fitted with HAs are key to making appropriate recommendations. The first 3 years of life are essential for acquiring a spoken language. During this time, the auditory system perceives speech signals in the environment and transmits them to specific areas of the brain, thus saving the development of head-to-head communication skills. Theoretically, it is also the best age window for children to receive implants [3, 4]. As the tools to measure speech and language development objectively in Mandarin-speaking children aged <3 years are very limited, making recommendations without missing the optimal implantation age based on limited data are clinically challenging.

The administration of open-set speech perception tests is not possible for children aged <3. Therefore, early speech perception (ESP) information in young children is mainly derived from the closed-set test. The Mandarin Early Speech Perception (MESP) test is a closed-set measure of speech perception tasks using words; it is the only test available to assess speech perception of Mandarin-speaking children as young as 2 years of age [5]. The MESP test was developed based on the English ESP test [6]. Due to the differences between Mandarin and English, only the first three categories (speech sound detection, speech pattern, and spondee perception) are similar between the MESP test and the English ESP test, and category 4 of the English ESP test, which includes 12 monosyllabic words, was revised to form categories 4 (vowel perception), 5 (consonant perception), and 6 (tone perception) of the MESP test. The two languages differ greatly in terms of syllables, stress patterns, vowels, and consonants. Most Mandarin syllables comprise three parts: an initial consonant, a syllable vowel, and a tone. Mandarin uses tone or pitch variations to convey lexical information, unlike Western languages. Therefore, assessment of tone perception is essential when evaluating Mandarin monosyllabic word recognition.

In the past 10 years, many studies have reported on the development of early speech perception in children with normal hearing and children with CIs [5, 7–16]. Unfortunately, the development of early speech perception in Mandarin-speaking children with HAs remains unexplored. Certainly, theoretically speaking, children with severe HL fitted with HAs can be considered implantation candidates if their speech perception lags behind that of those with CIs. However, many studies have shown concern about the ability of current CI speech processors to provide cues for the acquisition of Mandarin, and the results of most studies have shown that tone perception is challenging for Mandarin-speaking children with CIs [7, 9, 11–14]. In these studies, the accuracy of tone perception in Mandarin-speaking children with CIs was <80% regardless of the age at the time of implantation and the duration of CI use. It is well known that the basic working principles of HAs and CIs are different. HA amplifies the sound and senses it through the user's own hair cells. CIs bypass the damaged hair cells and sense sound directly by stimulating the auditory nerve and converting the sound into electrical stimulation. Suppose there is an objective gap between CIs and HAs in improving tone perception in children with HL. In that case, tone perception results will not be suitable as a data reference for identifying candidates for CIs.

The current research aimed to examine the development of speech perception of Mandarin monosyllabic words using the MESP test in children with severe HL fitted with HAs before 3 years of age. To avoid the impact on speech perception due to insufficient auditory compensation [2, 17], this study selected children with severe HL whose degree of HL ranged from 60 to 70 dB·HL in the better ear as the subjects.

## 2. Materials and Methods

### 2.1. Design and Sampling

This study comprised 95 children from the Department of Otolaryngology, Head and Neck Surgery Hearing Center at West China Hospital of Sichuan University. The inclusion criteria were as follows: children with the pure tone average (PTA, at 0.5, 1, 2, and 4 kHz) of the better ear ranging from 60 to 70 dB·HL; children who were fitted bilaterally with HAs before the age of 3 years; children with no other known developmental disabilities; children with parents and caregivers who were native speakers of Mandarin; and children with speech being the main mode of communication within their families. The exclusion criteria were as follows: children with a history of otorhinolaryngological surgery; children who abandoned the treatment; children who received CIs; children with the presence of syndromes (e.g., Down's syndrome) and associated neurological alterations; and children with other developmental abnormalities. The study protocol was approved by the medical ethics committee of our hospital, and written informed consent was obtained from the children's parents. All patients in this study completed this study, and no one dropped out of the study.

The age and gender distribution for the sample are shown in Table 1. The mean unaided PTA in the better ear for all subjects was 64.8 dB HL (SD = 3.4), and the aided PTA was 25.1 dB HL (SD = 5.4). The average duration of daily HA use was over 10 h for each age group. Subjects were assessed at 12, 24, and 36 months after fitting.  Table 2 shows the number of children who participated in each assessment. Based on the fitted age, the samples were stratified at 12 months as an interval, allowing for analysis of assessment data for each age group. Stratification for the current study comprised three groups based on the age at the time of fitting: <1 , 1–2, and 2–3 years. Since the minimum age of a child for using existing Mandarin speech perception materials is 2 years and children aged <1 years could not reach the assessment age until 2 years after fitting, the speech perception of children aged <1 year was reported only at the second and third year after fitting.

### 2.2. Speech Perception Assessment

Zheng et al. developed the MESP test [5], which is a tool commonly used to measure the earliest evidence of speech perception in a child for standard Mandarin. Zheng et al. [5] and Zhang et al. [16] used the MESP test to study the speech perception ability of children with normal hearing and established normal reference values. The MESP test has successfully evaluated early speech perception development in young Mandarin-speaking children after cochlear implantation [8, 10, 12–15]. This test includes the following six hierarchical categories of speech perception with increasing difficulty levels: 1: speech sound detection; 2: speech pattern; 3: spondee perception; 4: vowel perception; 5: consonant perception; and 6: tone perception. All the test words were presented in the form of pictures. Category 1 is used only to determine whether the subject can perform the MESP test, and no scores are calculated. Each of the categories 2–5 comprises only one test picture, and each picture has 12 test words. In category 6 (tone perception), there are six pictures because there are four tones in standard Mandarin, and six tone pairs can be formed. Each picture includes eight test words.

The MESP test software captured every response on every trial and used the responses to determine the overall speech perception of each individual. All these test results were presented in percentages. Since each measure was obtained from a closed set of response alternatives, the chance performance level and threshold scores required for significance above chance (*P* < 0.05) for each measure were used in the analyses. The percentages of the threshold scores for speech pattern, spondee, vowel, and consonant perception were 54.5%, 30.3%, 63.6%, and 63.6%, respectively. The threshold scores for overall tone perception, individual tone pair discrimination, and individual tone recognition were 68.3%, 75.0%, and 67.5%, respectively. As the categories advanced, the children not meeting a threshold score were dropped out from being tested for the next, more challenging category.  Table 2 displays the percentage of the sample from each age group that reached each category as well as the percentage with scores significantly better than chance.

### 2.3. Data Analyses

The data analysis focused on determining (1) the percentage of subjects whose performance scores were significantly above the threshold scores for each category, (2) the mean scores for each category, and (3) the accuracy of discriminating each of the six tone pairs and recognizing each of the four individual tones. Note that the mean scores are from the subjects whose scores were significantly above the threshold scores. The MESP test scores were compared for the present participants and their normal-hearing peers. A *P*-value of <0.05 was considered significant.

## 3. Results

### 3.1. Category 2: Speech Pattern Perception

Although the percentage of children who scored significantly above the threshold score improved from 84.2% (2–3 years group) and 86.4% (1–2 years group) at 12 months after fitting to 100% (both groups) at 36 months after fitting, the improvement was statistically not significant (*P* > 0.05). Category 2 scores of children in all age groups were above the threshold score after 2 years of HA use (Table 2). When a child's score was higher than the threshold score of category 2, the child was considered to have achieved category 2.

The mean scores for category 2 in each age group for every test interval are shown in Figure 1(a). This category seemed easy for the children as the mean score of 1–2 and 2–3 years groups at 12 months after fitting showed >90.0% accuracy. The improvement from 12 to 36 months after fitting was not significant in any age group (*P* > 0.05), and the age at the time of fitting did not significantly influence the performance of children in category 2 (*P* > 0.05).

### 3.2. Category 3: Spondee Perception

The results for category 3 are similar to those for category 2. Although the percentage of children who scored significantly above the threshold score improved from 87.0% (1–2 years group) and 88.2% (2–3 years group) at 12 months after fitting to 100% (both groups) at 36 months after fitting, the improvement was statistically not significant (*P* > 0.05). Category 3 scores of children in all age groups were above the threshold score after 2 years of HA use (Table 2). The mean score of the 1–2  and 2–3 years groups revealed an accuracy of >94.0% at 12 months after fitting (Figure 1(b)). The improvement from 12 to 36 months after fitting was not significant in any age group (*P* > 0.05), and the age at the time of fitting did not significantly influence the performance of children in category 3 (*P* > 0.05).

Previously, Zheng et al. [5] reported that all children with normal hearing successfully achieved categories 2 and 3, and the scores of children with normal hearing aged 2–3 years in categories 2 and 3 were 99.4%, and 100.0%, respectively. Therefore, our results indicate that children with severe HL can achieve better speech pattern and spondee perception after 12 months of HA use and that the age minimally influences the performance in these two categories at the fitting time.

### 3.3. Category 4: Vowel Perception

The percentage of children who scored significantly above the threshold score improved significantly from 47.1% (1–2 years group) and 43.7% (2–3 years group) at 12 months after fitting to 91.7% (<1 year group), 92.3% (1–2 years group), and 100% (2–3 years) at 36 months after fitting (*P* < 0.05; Table 2). The mean score of the three age groups significantly improved from 75.0% (1–2 years group) and 77.0% (2–3 years group) at 12 months after fitting to 84.8% (<1 year group), 85.3% (1–2 years group), and 88.1% (2–3 years group) at 36 months after fitting (*P* < 0.05; Figure 1(c)). For 1–2 and 2–3 years groups, the scores at 12 months after fitting were significantly different from those at 24 and 36 months after fitting, and the scores at 24 months after fitting were significantly different from those at 36 months after fitting (*P* < 0.05). For <1 year group, the scores at 24 months after fitting were significantly different from those at 36 months after fitting (*P* < 0.05). However, the differences among the three age groups at the same evaluation interval were insignificant (*P* > 0.05). The average score of children with normal hearing aged 2–3 years in category 4 was 90.8% [5]. Thus, after 36 months of HA use, the vowel perception of children with severe HL fitted with HAs before 3 years of age was comparable to that of children with normal hearing aged 2–3 years.

### 3.4. Category 5: Consonant Perception

The percentage of children who scored significantly above the threshold score improved significantly from 52.9% (1–2 years group) and 56.3% (2–3 years group) at 12 months after fitting to 94.2% (<1 year group), 92.3% (1–2 years group), and 91.6% (2–3 years group) at 36 months after fitting (*P* < 0.05; Table 2). The mean score of the three age groups improved significantly from 83.5% (1–2 years group) and 82.0% (2–3 years group) at 12 months after fitting to 89.0% (<1 year group), 89.7% (1–2 years group), and 89.5% (2–3 years group) at 36 months after fitting (*P* < 0.05; Figure 1(d)). For all age groups, the improvement from 24 to 36 months was not significant (*P* > 0.05). For 1–2  and 2–3 years groups, there was a significant improvement from 12 to 36 months after fitting (*P* < 0.05). However, the difference among the three age groups at the same evaluation interval was insignificant (*P* > 0.05). The average score of children with normal hearing aged 2–3 years in category 5 was 90.1% [5]. Thus, after 36 months of HA use, the consonant perception of children with severe HL fitted with HAs before 3 years of age was comparable to that of children with normal hearing aged 2–3 years.

### 3.5. Category 6: Tone Perception

The percentage of children who scored significantly above the threshold score improved significantly from 41.2% (1–2 years) and 43.8% (2–3 years) at 12 months after fitting to 91.2% (<1 year group), 92.3% (1–2 years group), and 91.6 (2–3 years group) at 36 months after fitting (*P* < 0.05; Table 2). The mean score of the three age groups improved significantly from 76.0% (1–2 years group) and 79.0% (2–3 years group) at 12 months after fitting to 87.6% (<1 year group), 87.7% (1–2 years group), and 88.9% (2–3 years group) at 36 months after fitting (*P* < 0.05; Figure 1(e)). For the 1–2  and 2–3 years groups, the scores at 12 months after fitting were significantly different from those at 24 and 36 months after fitting, and the scores at 24 months after fitting were significantly different from those at 36 months after fitting (*P* < 0.05). For the <1 year group, the scores at 24 months after fitting were significantly different from those at 36 months after fitting (*P* < 0.05). However, the difference among the three age groups at the same evaluation interval was not significant (*P* > 0.05). In category 6, the average score was 79.3% for children with normal hearing aged 2–3 years, 84.7% for those aged 3–4 years, and 90.6% for those aged 4–5 years [16]. The mean score of children in the <1 year group in the present study was higher than that of age-matched children with normal hearing reported by Zhang et al. [16]. For 1–2  and 2–3 years groups, the mean score at 12 months after fitting was comparable to that of children with normal hearing aged 2–3 years. Furthermore, the mean score at 24 months after fitting was comparable to that of children with normal hearing aged 3–4 years, and the mean score at 36 months after fitting was comparable to that of children with normal hearing aged 4–5 years.

### 3.6. Tone Pair Discrimination

For each of the six tone pairs, the mean percent correct discrimination scores of children at different test intervals for the three age groups are shown in Figure 2. For the < 1 year group (Figure 2(a)), the scores for only tone pair 1–4 improved significantly from 24 to 36 months after fitting (*P* < 0.05). For the 1–2 years group (Figure 2(b)), the scores for tone pairs 1–2 and 1–3 improved significantly from 12 to 24 months after fitting (*P* < 0.05). The scores for only tone pair 2–3 improved significantly from 24 to 36 months after fitting (*P* < 0.05). Finally, the scores for tone pairs 1–2, 2–3, and 2–4 improved significantly from 12 to 36 months after fitting (*P* < 0.05). For the 2–3 years group (Figure 2(c)), the scores for tone pairs 1–2 and 3–4 improved significantly from 12 to 24 months after fitting. The scores for only tone pairs 2–3 significantly enhanced from 24 to 36 months after fitting (*P* < 0.05). Finally, the scores for tone pairs 1–3, 1–4, 2–3, and 3–4 improved significantly from 12 to 36 months after fitting (*P* < 0.05). Notably, the scores for tone pair 2–3 did not exceed chance performance levels even at 36 months after fitting in any age group.

### 3.7. Tone Recognition

For each of the four tones, the mean percent correct recognition scores of children at different test intervals for the three age groups are shown in Figure 3. For the <1 year group (Figure 3(a)), the scores for tones 2 and 3 improved significantly from 24 to 36 months after fitting (*P* < 0.05). For the 1–2 years group (Figure 3(b)), the scores for tones 1 and 3 improved significantly from 12 to 24 months after fitting (*P* < 0.05). None of the tones' scores improved significantly from 24 to 36 months after fitting (*P* > 0.05). Finally, the scores for tones 1, 3, and 4 improved significantly from 12 to 36 months after fitting (*P* < 0.05). For the 2–3 years group (Figure 3(c)), the scores for only tone 3 improved significantly from 12 to 24 months after fitting (*P* < 0.05). None of the tones' scores improved significantly from 24 to 36 months after fitting. Finally (*P* > 0.05), the scores for tones 2 and 3 improved significantly from 12 to 36 months after fitting (*P* < 0.05). Notably, the scores for tone 3 in 1–2  and 2–3 years groups did not exceed chance performance levels even at 12 months after fitting.

## 4. Discussion

The main purpose of this study was to investigate early speech perception in Mandarin-speaking children with severe HL who had been fitted with HAs before the age of 3 years. The speech perception skills of these children significantly improved during the first 36 months of HA use, particularly for the aspects of vowel, consonant, and tone perception. The three age groups exhibited similar patterns of speech perception development. Although the three age groups showed similar trajectories of speech perception, the earlier intervention was associated with a smaller developmental gap between children with severe HL and age-matched children with normal hearing.

In the current study, Mandarin-speaking children with HA had significant improvements in speech perception. When comparing the speech perception performance of children with HAs and children with normal hearing [5], a very large gap in speech perception between the two was noted during the first year after fitting. This gap gradually narrowed with the increased duration of HA use. Zheng et al. [5] established the MESP test by investigating 2- to 5-year-old children with normal hearing (*N* = 92); they reported that all children successfully achieved categories 2–5 by 2 years of age; they performed equally well in categories 2–5, and their mean scores in these categories exceeded 90%. All children successfully achieved category 6 by 3 years of age, and their mean scores in this category approached 90%. In the current study, over 80% of subjects achieved categories 2 and 3 at 12 months after fitting, whereas nearly half of the subjects did not achieve categories 4, 5, and 6 over the same period. At 24 months after fitting, all subjects achieved categories 2 and 3. At 36 months after fitting, over 90% of subjects in the three age groups achieved categories 4, 5, and 6. The mean scores in categories 2 and 3 exceeded 90% at 12 months after fitting, whereas the mean scores in categories 4, 5, and 6 approached 90% at 36 months after fitting, regardless of the age at the time of fitting. Speech pattern and spondee perception subtests were evidently easy for children with HAs. As these two categories are designed for children with profound HL, the focus is on subjects' identification of lexical rhythms rather than on recognizing true monosyllabic words [5]. However, vowel, consonant, and tone perception results suggested that children with severe HL found it challenging to acquire the perception of Mandarin monosyllabic words in these aspects. We noted that most children with severe HL needed at least 36 months of HA use to acquire good vowel, consonant, and tone perception of Mandarin monosyllabic words.

Acquiring the ability to recognize monosyllabic words is similarly challenging for children with CIs [8, 13, 15, 18]. For example, Lu et al. [15] used the MESP test to report speech perception developments in 132 children who received CIs between the ages of 8 months and 7 years during the 24 months after receiving CIs. The results showed that <50% of pediatric CI users achieved tone perception category within the first year of implantation, and 70% of subjects achieved tone perception category 2 years after implantation. Eisenberg et al. [18] used the English version of the ESP test and reported that 20/42 children (48.0%) who received an implant at 2.3 years of age achieved category 4 (monosyllabic word identification) within the first year after implantation. However, Baumgartner et al. [19] investigated the speech perception performance of 33 German-speaking children with CIs during 36 months after implantation and found that the scores of the closed-set monosyllabic word tests were 100% at 12 months after implantation and remained steady over the 36-month evaluation period. This suggests that the process of monosyllabic word perception differs among children with HL belonging to different language backgrounds.

Although vowel, consonant, and tone perception subtests evaluate segmental perception of Mandarin monosyllabic words, the tone perception subtest is more challenging for children with normal hearing [5]. Zhang et al. [16] found that tone perception ability in children with normal hearing continues to develop from 2 to 6 years of age. However, children with severe HL performed equally well on vowel, consonant, and tone perception at each test interval. In the present study, children with HAs performed as well as or better than children with normal hearing in the tone perception subtest. For the 1–2  and 2–3 years groups, the mean tone perception scores were 76% and 79% at 12 months after fitting, respectively, which show that these children performed as well as 2-year-old children with normal hearing [16]. The mean tone perception score for the < 1 year group was 82.1% at 24 months after fitting, indicating better performance than that of 2-year-old children with normal hearing. Meanwhile, the patterns of tone pair discrimination and tone identification for children with HAs in the current study were similar to those of children with normal hearing [5, 16]. The mean score for tone pairs 2–3 at each test interval was significantly lower than that for other tone pairs in all three age groups. This may be because tones 2 and 3 have similar characterizations of tone height; tone 2 has a rising contour and tone 3 has a falling dip and then a rising contour, therefore, tones 2 and 3 show similar rising contours [16]. It can be inferred that children with severe HL fitted with HAs can rapidly acquire tone perception in the early stage of speech development, and the duration of HA use was a significant predictor of tone perception.

A review of previous studies on tone perception in children with CIs found that the mean score of tone perception did not exceed 80%, except in case reports. For example, Peng et al. [7] reported the tone perception of 30 children who received CIs at 5.8 years of age and had used CIs for 3.7 years, and results showed that the mean score of tone perception was 72.9%. Xu et al. [9] reported that the mean score of tone perception was 71.0% in 25 children who received CIs at 6.4 years of age and had used them for 3.1 years. Zhou et al. [11] investigated the tone perception ability of 110 children with CIs at 3.9 years of age who had used them for 1.3 years. The results showed that the mean score of tone perception was 67.3%. Chen et al. [12] used the MESP test to evaluate tone perception in children who received implants at the age of 2.7 years and whose duration of CI use was 1.5 years. The results showed that the mean score of tone perception was 77%. Li et al. [13] also used the MESP test to evaluate tone perception in 12 children who received implants at the age of 35 months, and the results showed that the mean score of tone perception was 79.9% after 3 years of CI use.

Recently, Li et al. [14] conducted a retrospective cross-sectional study that also used the MESP test to evaluate the development of tone perception during the 48 months after implantation in children who received the implant at 1–4 years of age. The tone perception scores ranged from 70% to 80% for all age groups, and neither the age at the time of implantation nor the duration of CI use was significantly related to the tone perception score. In all of the above studies, the scores of tone perception showed great individual differences, and the scores ranged from near-chance-level scores to near-perfect scores. However, regarding the mean scores of tone perception, children with severe HL fitted with HAs in the present study performed better than children with CIs in previous studies.

There are also some shortcomings in this study. The patients in this study are all from the same hospital, not representative of the overall level, and sample size of this study is small; these problems can lead to some bias in the results of this study.

## 5. Conclusions

Our findings provide the first evidence that HAs can effectively promote the development of speech perception in Mandarin-speaking children with severe HL. The developmental trajectories of speech perception after fitting were similar for children who were fitted with HAs within 3 years of age. Furthermore, HAs can synchronously improve their vowel, consonant, and tone perception. Most Mandarin-speaking children with severe HL fitted with HAs can master speech pattern and spondee perception skills within 12 months of fitting Has, and master vowel, consonant, and tone perception within 36 months of fitting HAs. The outcomes of tone perception were better for children with HAs than for children with CIs reported in previous studies.

## Figures and Tables

**Figure 1:** The mean scores in categories 2–6 in three age groups at each test interval.

**Figure 2:** The mean scores for the discrimination of six tone pairs in three age groups at each test interval. The dashed line displays the threshold score for individual tone pair discrimination.

**Figure 3:** At each test interval, the mean scores for the recognition of four tones in three age groups. the dashed line displays the threshold score for individual tone recognition

**Table 1:** General characteristics of subjects.

Gender	Age at the time of fitting			Totals
	<1 year	1–2 years	2–3 years	
Male	22	14	12	48
Female	23	13	11	47
Total	45	27	23	95
Mean age	0.5	1.6	2.5	1.5
Percent of sample	47.4%	28.4%	24.2	100%

**Table 2:** The number of children who were tested in each category of the MESP test and the percentages of children who achieved each category.

Age at the time of fitting	<1 year		1–2 years			2–3 years		
	24 months	36 months	12 months	24 months	36 months	12 months	24 months	36 months
Number								
Category 2	42	38	23	18	14	19	14	12
Category 3	41	36	22	18	14	17	14	12
Category 4	37	36	19	15	13	16	13	12
Category 5	36	35	17	13	13	16	12	11
Category 6	35	34	17	12	13	15	11	11

Proportion (%)								
Category 2	100	100	86.4	100	100	84.2	100	100
Category 3	100	100	87	100	100	88.2	100	100
Category 4	86.5	91.7	47.1	80	92.3	43.7	92.3	100
Category 5	77.8	94.2	52.9	76.9	92.3	56.3	83.3	91.6
Category 6	77.1	91.2	41.2	83.3	92.3	43.8	81.8	91.6

## Data Availability

The datasets used and analyzed during the current study are available from the corresponding author upon reasonable request.
